# The Impact of Neutrophil-Lymphocyte Ratio in Febrile Seizures: A Systematic Review and Meta-Analysis

**DOI:** 10.1155/2022/8472795

**Published:** 2022-10-11

**Authors:** Samaneh Hosseini, Hossein Gharedaghi, Sina Hassannezhad, Shahram Sadeghvand, Amirhossein Maghari, Saeed Dastgiri, Mahnaz Talebi, Shokoufeh Khanzadeh

**Affiliations:** ^1^Neurosciences Research Center, Tabriz University of Medical Sciences, Tabriz, Iran; ^2^School of Medicine, Zanjan University of Medical Sciences, Zanjan, Iran; ^3^Cardiovascular Research Center, Tabriz University of Medical Sciences, Tabriz, Iran; ^4^Pediatric Health Research Center, Tabriz University of Medical Sciences, Tabriz, Iran; ^5^Department of Family Health, Social Determinants of Health Research Center (SDHRC), Ardabil University of Medical Sciences, Ardabil, Iran; ^6^Tabriz Health Services Management Research Center, Tabriz University of Medical Sciences, Tabriz, Iran; ^7^Neurosciences Research Center (NSRC), Tabriz University of Medical Sciences, Tabriz, Iran; ^8^Student Research Committee, Tabriz University of Medical Sciences, Tabriz, Iran

## Abstract

This meta-analysis was conducted to determine the relationship between neutrophil to lymphocyte ratio (NLR) and febrile seizure (FS). Our study was registered with the PROSPERO (ID: CRD42021259944). Web of Science, Embase, PubMed, Scopus, and ProQuest Central were searched, and finally, 17 studies were included. Standardized mean difference (SMD) was reported with a 95% confidence interval (CI) for the NLR levels. Compared with the febrile control group, the FS patients' NLR levels were significantly higher (SMD = 0.49; 95%CI = 0.26 to 0.72, *P* < 0.001). Furthermore, we conducted a comparison of NLR levels between febrile controls against simple and complex FS cases separately and found that NLR levels of children with either simple or complex FS were higher compared with those of febrile controls (SMD = 0.42, 95%CI = 0.14 to 0.69, *P* = 0.003 and SMD = 0.90, 95%CI = 0.71 to 1.09, *P* < 0.001, respectively). Also, in comparison with the NLR levels of the simple FS group, the complex FS patients' NLR levels were significantly higher (SMD = 0.59, 95%CI = 0.34 to 0.85, *P* < 0.001). Our study indicated that NLR could be recommended as an inexpensive diagnostic biomarker for FS. In addition, it can be useful when distinguishing between simple FS and complex FS.

## 1. Introduction

Febrile seizure (FS) is conceived as the most common type of childhood seizure, affecting about 2–5% of children under six years [1]. FS is defined as a rapidly rising or elevated body temperature accompanied by an uncomplicated seizure, with no history of neurologic abnormality, previous unprovoked seizure, and previous neonatal seizure, and does not meet the diagnostic criteria for other acute symptomatic seizures and not predisposed to subsequent epilepsy, in children aged six months to five years [1, 2]. FS can be classified into two groups: complex FS lasts ≥15 min, is focal, and recurs within 24 h, while simple FS lasts <15 min, only occurs once in 24 h, and is generalized [1].

Although fever is a prevalent symptom in childhood, it is accompanied by subsequent seizures only in a few children, and it is not yet clear how fever can irritate the brain and generates FS2. However, research has consistently suggested that inflammatory pathways intrinsic to the febrile response can explain susceptibility to seizures in such febrile children [2]. Accordingly, inflammatory cytokines, particularly TNF-*α*, interleukin- (IL-) 6, and IL-1*β*, are the most extensively used biomarkers for the inflammation status in children with FS [3]. However, a major problem with these kinds of cytokines is their limited availability; so several attempts have been made to discover some available and inexpensive markers to determine the inflammatory response status in such patients. Recent evidence suggests that neutrophil to lymphocyte ratio (NLR) may be used as an available and inexpensive marker for systemic inflammation, given the role of inflammatory pathways in the hematopoietic multiple-lineage changes [4]. The NLR, which can be calculated by absolute neutrophil count divided by absolute lymphocyte count, assessed based on a complete blood count (CBC) differential test, has been investigated in a number of previous studies involving cardiovascular diseases, malignancies [5, 6], and some neurologic disorders [7]; however, the relevance between NLR and FS is still unclear. Although the controversy about the association between NLR and FS has raged unabated for about a decade [8–24], no systematic review has been reported. Therefore, our systematic review was conducted to determine whether NLR is associated with FS susceptibility and FS types in children. A better knowledge of the link between NLR and FS will assist in elucidating the role of inflammation and immunology in the progression and prognosis of this condition, as well as identify patients who require early intervention and further monitoring and imaging; so the results of this study can serve to validate NLR as emerging biomarkers for FS while simultaneously elucidating pathophysiology to potentiate therapeutic development.

## 2. Materials and Methods

### 2.1. Protocol and Registration

Our study was registered with the PROSPERO (ID: CRD42021259944).

### 2.2. Search Strategy

We conducted a systematic review and meta-analysis to retrieve all published documents, including preprints and grey literature, in accordance with Preferred Reporting Items for Systematic Review and Meta-analyses (PRISMA) guidelines (Figure 1).

Two reviewers (Sh.Kh., A.M.) performed a systematic literature search in the online databases of Web of Science, Embase, PubMed, Scopus, and ProQuest Central, independently.

The last update of the search was conducted on June 28, 2021. Our search strategy was not restricted by language or year of publication. The reference lists of relevant reviews and articles were also interrogated to identify potentially eligible studies. Also, Prospero Register was searched for details of unpublished and ongoing studies. To identify grey literature and further relevant studies, we also conducted a quick nonsystematic search in Google Scholar as a secondary database in English, Chinese, and Turkish because the majority of identified articles were conducted in China and Turkey.

### 2.3. Inclusion and Exclusion Criteria

The inclusion criteria were as follows: (1) cross-sectional, nested case-control, or case-control studies comparing the value of NLR between children (aged between 5 to 72 months) with FS and those with fever but no seizures or children with simple seizure and those with complex seizure. (2) It reported adequate and informative data, including the number of subjects in both the control and the case groups and the mean and standard deviation of NLR in both the control and case groups needed to estimate the weighted mean difference.

The exclusion criteria were as follows: (1) studies in which the control group consisted of healthy subjects; (2) studies that enrolled subjects with any concomitant disorders such as meningitis; (3) animal studies, letters to editors, case series, and case reports; (4) randomized controlled trials and cohort studies because such studies have not yet been reported; (5) studies with overlapping data; and (6) duplicated studies.

### 2.4. Data Extraction and Quality Assessment

The titles/abstracts of the obtained articles were investigated by two authors (SH.KH. and M.T.) separately. Then, the same two authors independently checked the full texts of relevant articles for eligibility. Any discrepancies between reviewers in both steps were resolved by a third independent author (S.D.).

The extracted data were as follows: the type of document (article or dissertation), the first author, year of publication, language, study location, ethnicity, study design, age group (months), total sample size as well as the number of simple and complex FS cases and controls separately, percentage of males among FS cases, the percentage of patients with the previous history of FS, mean ± SD of NLR level in cases (all cases, simple FS, and complex FS) and controls, or sufficient data for estimating the mean ± SD such as median and interquartile range (IQR) or/and range. In the case of discrepancies, the consensus was obtained after discussion with a third author (S.D.).

An assessment of the quality of included studies was performed by two authors (Sh.Kh. and M.T.) independently based on the Newcastle-Ottawa Scale, which comprises three sections: selection (4 items), comparability (2 items), and exposure (3 items), with a total score of 0 to 9. Any disagreements were finally reconciled through arbitration by a third author (S.D.).

### 2.5. Statistical Analysis

Standardized mean difference (SMD) was reported with a 95% confidence interval (CI) for the NLR level. Calculating the mean and SD from the median, sample size and range, and/or IQR was performed using the methods introduced by Wan et al. [25]. Heterogeneity between study results was assessed by the chi-squared (*χ*^2^) test and *I*^2^ statistic: the *χ*^2^ test was applied to the evaluation of whether heterogeneity is present, and the *I*^2^ statistic was applied to quantify inconsistency across studies: *I*^2^˃75% and *Pχ*^2^ test ˂ 0.05 were considered as significant heterogeneity of results. In such a case, the source of heterogeneity was investigated based on several methods: metaregression tests, subgroup analysis, and exclusion of each study one at a time to assess the effect of each study. Also, a random-effects model was adopted for the meta-analysis of heterogeneous results. Otherwise, we used the fixed-effect model. For detection of potential publication bias, Egger's linear-regression test and funnel plot were applied, and those with a *P* value of ˂0.05 were conceived to have significant publication bias. STATA 12.0 software (Stata Corporation, College Station, TX, USA) was applied for statistical analyses. A *P* value ≤ 0.05 was conceived as statistically significant.

## 3. Results

### 3.1. Literature Search and Selection

Figure 1 shows the process of identifying and selecting research evidence in this systematic review. In addition to 318 studies from the initial database search, eight further studies identified through reference lists of relevant articles and search in Google Scholar were added. After removing duplicates, the titles and abstracts of 290 remaining studies were reviewed, and 23 studies were selected for full-text review. Then, six studies were excluded (the reasons for exclusion are clarified in Figure 1), and finally, 17 studies were included in the present meta-analysis.

### 3.2. Characteristics of the Included Studies

Of the 17 studies included in this meta-analysis, six studies were retrospective cross-sectional [9, 10, 12, 14, 19, 21], ten studies were retrospective case-controlled [8, 11, 13, 15–17, 20, 22–24], and one study was prospective case-controlled [18]. With respect to document language, there were 13 documents in English [8, 11–22], 3 in Chinese [10, 23, 24], and 1 in Turkish [9]. In regard to document type, there were 16 articles [8, 10–24] and one doctoral dissertation [9]. Overall, 1079 controls and 1919 FS children were enrolled in the selected studies. The general characteristics of the selected studies are presented in Table 1. Although the quality assessment of selected studies assessed with the Newcastle-Ottawa Scale left different scores ranging from 4 to 9, we included all of them in the meta-analysis (Table 2).

Of the 17 studies, ten studies reported NLR levels in children with FS and compared them with that of controls [8, 11, 13, 15–18, 20, 22, 24], and 11 studies compared the NLR levels in children with simple FS with those of children with complex ^FS^ [8–10, 12–14, 16, 19–21, 23].

### 3.3. Meta-Analysis of Differences between FS Patients and Febrile Controls in NLR Level

NLR levels in FS children were compared with those of controls with the febrile disease without a seizure in 10 case-control studies with 1055 patients with FS and 1079 febrile controls. Compared with the control group, the FS patients' NLR levels were significantly higher (SMD = 0.49;  95%CI = 0.26 to 0.72, *P* < 0.001). The included studies were statistically heterogeneous (*I*^2^ = 80.4%, *P* heterogeneity < 0.001). Thus, the random-effects model was used for the meta-analysis (Figure 2). In addition, when we included the sample size as a covariate in a metaregression model, we found that the sample size significantly affected the SMD (*P* value = 0.033). So it may be a potential source of heterogeneity in our meta-analysis. Interestingly, classification of studies into two subgroups of small (sample size ≤ 210) and large studies (sample size > 210) left a relatively little heterogeneity between studies. However, in both subgroups, the NLR levels of FS patients were significantly higher than those of controls (SMD = 0.33, 95%CI = 0.16-0.50, *P* value < 0.001, *I*^2^ = 44.5%, *P* heterogeneity = 0.094 in small studies vs. SMD = 0.87, 95%CI = 0.71-1.03, *P* value < 0.001, *I*^2^ = 38.1%*P* heterogeneity = 0.119 in large studies) (Figure 3).

In another subgroup analysis according to whether the participants developed their first FSs or subsequent FSs, there were two studies, including solely the participants without previous history of FS; they included 445 patients with FS and 445 febrile controls. The remaining six studies compared controls and FS patients irrespective of the number of previous seizures. The NLR levels in children with first FS were significantly more than in febrile children (SMD = 0.84, 95%CI = 0.63 to 1.05, *P* value < 0.001) (Figure 4).

In the third subgroup analysis, we classified studies according to the ethnicity of participants. There were three studies of participants of Asian ethnicity, including 404 FS children and 410 febrile controls. Compared with the control group's NLR levels, the Asian patient group's SMD was 0.693 (95%CI = 0.369 to 1.018, *P* value < 0.001). There were four studies of participants of Caucasian ethnicity; they included 315 patients with FS and 343 febrile controls. Compared with the control group's NLR levels, the Caucasian patient group's SMD was 0.32 (95%CI = 0.14 to 0.49, *P* value = 0.001).

Two investigations examined Indian participants and included 296 patients with FS and 296 febrile controls and reported lower NLR levels in FS children than in febrile children. However, it was not statistically significant (SMD = 0.82, 95%CI = 0.53 to 1.12, *P* value < 0.001). Also, one study investigated Arab participants, including 40 FS patients and 30 febrile controls. Compared with the controls, the Arab patients' SMD was -0.01 (95%CI = −0.48 to 0.47, *P* value = 0.976) (Figure 5).

In the next step, we compared NLR levels between febrile controls against simple and complex FS cases separately based on studies for whom the data (NLR level and the number of simple and complex cases and controls) was available. Five studies, including 419 simple FS cases and 576 controls, had sufficient data for comparing the simple FS cases with controls, and four studies, including 184 complex FS cases and 498 controls, reported data needed for comparing complex FS cases with controls. Children with FS had significantly elevated levels of NLR compared with febrile controls, in either simple or complex FS group (SMD = 0.42, 95%CI = 0.14 to 0.69, *P* value = 0.003 and SMD = 0.90, 95%CI = 0.71 to 1.09, *P* value < 0.001, respectively) (Figure 6).

### 3.4. Meta-Analysis of Difference between Children with Simple and Complex FS in NLR Levels

NLR levels in simple FS children were compared with those of complex FS in 11 studies, of which four were case-controlled and six were cross-sectional, including 1363 patients with simple FSs and 460 patients with complex FS. In comparison with the simple FS group, the complex FS patients' NLR levels were significantly higher (SMD = 0.59, 95%CI = 0.34 to 0.85, *P* value < 0.001). The included studies were statistically heterogeneous (*I*^2^ = 75.9%, *P* heterogeneity < 0.001); thus, the random-effects model was applied for the meta-analysis (Figure 7). Metaregression gave no indication that heterogeneity between studies was attributable to the age of simple FS cases (*P* value = 0.55) and complex FS cases (*P* value = 0.48), ethnicity (*P* value = 0.92), design of the study (*P* value = 0.99), and the percentage of males (*P* value = 0.08). However, when we included the sample size as a covariate in a metaregression model, we found that SMD was affected by the sample size (*P* value = 0.05); so it may be a potential source of heterogeneity in our meta-analysis. Interestingly, classification of studies into three subgroups of small (sample size ≤ 100), medium (100˂sample size ≤ 200), and large studies (sample size > 200) left a relatively little heterogeneity between studies (Figure 8). In studies with small and medium sample size, the NLR levels of complex FS patients were significantly higher than those of simple FS cases (SMD = 0.73, 95%CI = 0.04-1.06, *P* value < 0.001 in small studies; SMD = 0.72, 95%CI = 0.41-1.04, *P* value < 0.001 in medium studies). However, in large studies, the simple and complex FS cases did not differ in NLR levels (SMD = 0.11, 95%CI = −0.32-0.54, *P* value = 0.60). Another possible reason for high heterogeneity is revealed in Figure 7. There were no differences in the results of different studies according to whether the NLR levels were higher in simple FS children or complex FS children, except for Kubota et al.'s study, which reported lower levels of NLR in children with complex FS compared with those with simple FS, although it was not statistically significant. When we excluded Kubota et al.'s study, heterogeneity was reduced to 58.6%(*P* heterogeneity = 0.010) between the remaining studies. The reason probably was that in the mentioned study, the levels of NLR in simple and complex FS groups were reported as median and IQR, and we estimated the mean and standard deviation using statistical methods; so the different results of the mentioned study may be attributed to some serious limitations of statistical methods for mean and standard deviation estimation.

In subgroup meta-analysis according to ethnicity, there were 6 studies on Caucasian participants (475 simple FS cases, 159 complex FS cases), 4 studies on Asian participants (412 simple FS cases, 217 complex FS cases), and one study on Indian subjects (46 simple FS cases, 54 complex FS cases) (Figure 9). Both Caucasian and Asian participants with complex FS showed more levels of NLR compared with those with simple FS (SMD = 0.68, 95%CI = 0.45-0.92, *P* value < 0.001 and SMD = 0.57, 95%CI = 0.02-1.12, *P* value = 0.042, respectively). Vice versa, in Indian patients' group, there was no significant difference between cases and controls (SMD = 0.32, 95%CI = −0.07 to 0.72, *P* value = 0.110).

In the second subgroup analysis, we identified five studies that included the participants solely without previous history of FS; they included 510 patients with simple FSs and 223 complex febrile children. The remaining five studies did not have such inclusion criteria. The NLR levels in simple FS children without previous history of FS were significantly more than those with complex FS (SMD = 0.59, 95%CI = 0.35-0.83, *P* value < 0.001) (Figure 10).

### 3.5. Publication Bias and Small Study Effect

As shown in Figure 11, the results of studies on differences in NLR levels between FS cases and febrile controls showed a statistically significant publication bias (Egger's test *P* value = 0.001). We identified two missing studies using Stata's metatrim command. After we included the missing studies in the meta-analysis, the NLR levels in FS cases were significantly higher than those of controls as before (SMD = 0.608, 95%CI = 0.373-0.843); therefore, reported publication bias was unlikely to influence the interpretation of our results. However, the results of studies that compared simple FS cases against complex FS cases indicated no evidence of publication bias. In addition, Egger's test revealed no statistically significant publication bias (*P* value = 0.156).

## 4. Discussion

Many recent studies have suggested that an elevated NLR is associated with febrile seizures [8–24]. Here, we undertook a meta-analysis of 17 studies comprising 1919 children with FS and 1079 febrile controls to assess the diagnostic role of NLR in FS. We found that children with FS had significantly elevated levels of NLR compared with febrile controls in either simple or complex FS groups. There are several possible explanations for these results, detailed below.

One potential mechanism explaining the high levels of NLR in FS patients is the role of inflammation in FSs [2]. A large and growing body of literature has shown that proinflammatory cytokines such as IL-1*β* and IL-6 and TNF-*α* were significantly higher in FS cases in either descriptive human studies or experimental studies [26, 27]. Moreover, it has been reported that high mobility group box 1 (HMGB1), which is a nuclear protein secreted from neutrophils, macrophages, and monocytes and triggers inflammation, increased in FS patients [26].

Although cytokines are the most used indicators for inflammation in exploring FS, a major concern with these markers is their unavailability and high cost. As a substitute, NLR is an objective, reproducible, low-cost, and available indicator of inflammation. It indicates the balance between two blood components: lymphocyte, the protective and regulatory component, and neutrophil, an important inflammatory component realizing proinflammatory products. There has been little discussion about the role of such cells in the context of FS patients [2, 26]; however, the increased levels of NLR in FS cases in our study reflected either increase in the neutrophil count or a decrease in lymphocyte count, suggesting that such cells contribute to the mechanisms that generate FS. The result of this study will now be compared to the findings of earlier studies. Lymphocytes have been shown to secrete IL-10, a multifunctional anti-inflammatory cytokine that increases the febrile seizure threshold, suggesting that lymphocyte function is associated with resistance to febrile seizures [2, 26]. Vice versa, neutrophils have been shown that act as an essential inflammatory component secreting and activating proinflammatory mediators attributed to increased seizure susceptibility such as HMGB1, IL-6, and IL-1*β* [2, 26]. So it is not surprising that increased NLR levels were found in FS patients compared with controls in our study.

Another possible explanation for our results is that iron deficiency anemia influences cell-mediated, humoral, and nonspecific immunity and is associated with an increased NLR [28]. Interestingly, it has been shown that the prevalence of iron deficiency anemia is higher among children with FS compared with healthy controls [29]. Further studies which take this condition as a confounding variable will need to be undertaken.

However, there are other possible explanations for our findings. These results could be attributed to the humoral system function [16]. Elevated cortisol levels reported during FSs due to sympathetic activation result in lymphopenia, neutrophilia, and leukocytosis [16]. It is not surprising, then, that the ratio of neutrophil to lymphocyte count (NLR) would increase.

Another important finding was that the complex FS patients' NLR levels were significantly higher in comparison with the simple FS group. Hence, it could conceivably be hypothesized that the level of inflammation in complex FS patients is higher than that of simple FS patients, and inflammation plays a more dominant role in the pathogenesis of complex FS than that of simple FS.

In combination, it seems that based on NLR levels, febrile children that would develop seizures could be distinguished from those that would not develop at an early stage after the febrile conditions. Furthermore, NLR could help physicians differentiate between simple FS and complex FS. Because both FS types require different management strategies and approaches, it is, therefore, crucial to identify the type of each FS. However, these findings cannot be extrapolated to all patients. In many FS patients, probably most, there is no need for a CBC test and exact NLR level since distinguishing between simple FS and complex FS was performed based on physical examination and taking a medical history from the parent [1]. But sometimes, differentiating between simple FS and complex FS can be confounding because of the change in clinical signs of the illness at admission, because of anticonvulsive therapy during patient transfer to hospital, as well as the insufficient anamnesis provided by the parent in an agitated condition [1]. So in case of a lack of reliable medical history or physical examination, NLR can help make an exact diagnosis. This combination of findings provides some support for the conceptual premise that anti-inflammatory drugs have therapeutic effects on seizures [30, 31]. This is an important issue for future research.

Although the study has successfully demonstrated that NLR has a strong association with FS, it has certain limitations. The main limitation of this study is the small number of papers that were included in the analysis. As such, our results may be limited in power, and additional studies would be warranted to strengthen the results of our study further. Furthermore, the studies included in our analysis exhibited high heterogeneity. Although this was accounted for with the random-effects model, such measures may not entirely eliminate the issue of heterogeneity. Nonetheless, our systematic search—in conjunction with a manual review of references from the resulting articles—has ensured a thorough and reliable search of the literature and serves as a notable strength of this study.

In conclusion, this meta-analysis indicated that NLR could be recommended as an inexpensive diagnostic biomarker for FS. In addition, it can be useful when distinguishing between simple FS and complex FS. However, further large high-quality investigations should be conducted to understand the relationship between inflammatory markers and FS better.

## Figures and Tables

**Figure 1:** Flowchart of search and study selection.

**Figure 2:** Meta-analysis of NLR levels in patients with FS and in febrile controls (random-effects model).

**Figure 3:** Subgroup meta-analysis of NLR levels in patients with FS and febrile controls (random-effects model) according to sample size.

**Figure 4:** Subgroup meta-analysis of NLR levels in patients with FS and febrile controls (random-effects model) according to the previous history of FS in participants.

**Figure 5:** Subgroup meta-analysis of NLR levels in patients with FS and febrile controls (random-effects model) according to ethnicity.

**Figure 6:** (a) Meta-analysis of NLR levels in patients with simple FS and febrile controls (random-effects model). (b) Meta-analysis of NLR levels in patients with complex FS and febrile controls (random-effects model).

**Figure 7:** Meta-analysis of NLR levels in patients with simple FS and patients with complex FS (random-effects model).

**Figure 8:** Subgroup meta-analysis of NLR levels in patients with simple FS and patients with complex FS (random-effects model) according to sample size.

**Figure 9:** Subgroup meta-analysis of NLR levels in patients with simple FS and patients with complex FS (random-effects model) according to ethnicity.

**Figure 10:** Subgroup meta-analysis of NLR levels in patients with simple FS and patients with complex FS (random-effects model) according to previous history of FS among participants.

**Figure 11:** Egger's test and funnel plot showing publication bias: (a) studies on NLR levels in patients with FS and febrile controls; (b) studies on NLR levels in patients with simple FS and patients with complex FS.

**Table 1:** General characteristic of the included studies.

First author	Publication year	Study design	Country/ethnicity	Age group (months)	Solely first FSs	Percentage of males among FS cases	FS cases						Febrile controls		NOS score
							All cases		Simple FS cases		Complex FS cases				
							Number	Mean ± SD of NLR	Number	Mean ± SD of NLR	Number	Mean ± SD of NLR	Number	Mean ± SD of NLR	
Goksugur, S.B.	2014	Cross-sectional	Turkey/Caucasian	6-70	Yes	61%	97	—	58	2.18 ± 1.91	39	3.89 ± 4.28	—	—	8
Yazar, A.	2018	Case control	Turkey/Caucasian	Not declared	No	52%	50	1.84 ± 1.82	39	1.43 ± 1.50	11	3.33 ± 2.14	49	1.91 ± 2.17	7
Yigit, Y.	2017	Cross-sectional	Turkey/Caucasian	6-60	Yes	51%	142	—	91	2.38 ± 1.60	51	3.42 ± 1.77	—	—	8
Gaoli, C.	2018	Cross-sectional	Chinese/Asian	6-60	No	50%	100	—	50	2.16 ± 1.26	50	—	—	—	6
Liu, Z.	2018	Case control	Chinese/Asian	5-72	Yes	69%	249	3.2 ± 2.4	167	2.9 ± 2.4	82	3.7 ± 2.5	249	1.6 ± 1.9	9
Balikoglu, P.	2019	Cross-sectional	Turkey/Caucasian	6-60	Yes	54%	112	—	89	2.06 ± 1.99	23	3.30 ± 3.81	—	—	8
Cokyaman, T.	2020	Case control	Turkey/Caucasian	5-72	No	51%	91	4.0 ± 4.28	—	—	—	—	116	2.6 ± 3.77	8
Khosravi, S.	2020	Case control	Iran/Caucasian	6-60	No	69%	100	3.066 ± 3.080	93	3.026 ± 3.093	7	3.600 ± 3.077	100	1.990 ± 2.669	5
Kubota, J.	2020	Cross-sectional	Japan/Asian	6-60	No	60%	205	4.17 ± 2.91	139	4.32 ± 2.97	66	3.98 ± 3.15	—	—	8
Liu, Z.	2020	Case control	Chinese/Asian	6-72	No	55%	75	—	56	2.43 ± 1.22	19	3.86 ± 1.36	—	—	4
Mhaibes, S.	2020	Case control	Iraq/Iraqi	6-60	No	62%	40	3.60 ± 2.72	—	—	—	—	30	3.62 ± 2.77	8
Moral, R.	2020	Case control	India/Indian	6-60	Yes	62%	196	2.06 ± 1.56	—	—	—	—	196	0.91 ± 0.78	5
Ornek, Z.	2020	Cross-sectional	Turkey/Caucasian	6-60	Yes	57%	133	—	105	3.80 ± 3.49	28	8.90 ± 8.12	—	—	8
Pooja, A.	2020	Case control	India/Indian	6-60	No	57%	100	4.5 ± 6.9	46	3.3 ± 4.0	84	5.5 ± 8.5	100	1.2 ± 1.8	4
Kurniawan, A.	2021	Case control	Indonesia/Asian	6-59	No	69%	52	4.73 ± 4.16	25	—	27	—	52	3.61 ± 3.92	6
Meiling, G.	2021	Case control	Chinese/Asian	6-60	No	59%	103	4.28 ± 0.57	—	—	—	—	109	3.72 ± 0.57	5
Yoldas, M.	2021	Case control	Turkey/Caucasian	6-60	No	56%	74	3.35 ± 8.1	74	3.35 ± 8.1	—	—	78	0.77 ± 0.67	7

**Table 2:** Risk of bias assessment of the included studies according to the modified Newcastle-Ottawa Scale (NOS).

NOS items	Goksugur, S.B.	Yazar, A.	Yigit, Y.	Gaoli, C.	Liu, Z. 2018	Balikoglu, P.	Cokyaman, T.	Khosravi, S.	Kubota, J.	Liu, Z. 2020	Mhaibes, S.	Moral, R.	Ornek, Z.	Pooja, A.	Kurniawan, A.	Meiling, G.	Yoldas, M.
Selection																	
Is the case definition adequate?	∗	∗	∗	•	∗	∗	∗	•	∗	•	∗	•	∗	•	•	•	∗
Representativeness of the cases	∗	∗	∗	•	∗	∗	•	•	∗	•	∗	•	∗	•	•	•	•
Selection of controls	∗	∗	∗	∗	∗	∗	∗	∗	∗	•	∗	•	∗	•	∗	•	∗
Definition of controls	∗	•	∗	∗	∗	∗	∗	∗	∗	•	∗	∗	∗	•	∗	∗	∗
Comparability																	
Study controls for the most important factor	∗	∗	∗	•	∗	•	∗	∗	∗	∗	∗	∗	∗	∗	•	∗	∗
Study controls for the second important factor	∗	∗	∗	∗	∗	∗	∗	•	∗	∗	∗	∗	∗	•	∗	∗	∗
Exposure																	
Was the measurement method of NLR described?	•	•	•	∗	∗	∗	∗	•	•	•	•	•	•	∗	∗	•	•
Were the methods of measurements similar for cases and controls?	∗	∗	∗	∗	∗	∗	∗	∗	∗	∗	∗	∗	∗	∗	∗	∗	∗
Nonresponse rate	∗	∗	∗	∗	∗	∗	∗	∗	∗	∗	∗	∗	∗	∗	∗	∗	∗
Total score	8	7	8	6	9	8	8	5	8	4	8	5	8	4	6	5	7

## Data Availability

The datasets generated during and/or analyzed during the current study are available from the corresponding author on reasonable request.
